The article "An Improved Stacked Autoencoder for Metabolomic Data Classification" was published in 2021. Journal: Comput Intell Neurosci.

# An Improved Stacked Autoencoder for Metabolomic Data Classification

**DOI:** 10.1155/2021/1051172

**Published:** 2021-08-15

**Authors:** Xiaojing Fan, Xiye Wang, Mingyang Jiang, Zhili Pei, Shicheng Qiao

**Affiliations:** ^1^College of Engineering, Inner Mongolia University for Nationalities, Tongliao 028000, China; ^2^College of Chemistry and Chemical Engineering, Inner Mongolia University for Nationalities, Tongliao 028000, China; ^3^College of Computer Science and Technology, Inner Mongolia University for Nationalities, Tongliao 028000, China

## Abstract

Naru3 (NR) is a traditional Mongolian medicine with high clinical efficacy and low incidence of side effects. Metabolomics is an approach that can facilitate the development of traditional drugs. However, metabolomic data have a high throughput, sparse, high-dimensional, and small sample nature, and their classification is challenging. Although deep learning methods have a wide range of applications, deep learning-based metabolomic studies have not been widely performed. We aimed to develop an improved stacked autoencoder (SAE) for metabolomic data classification. We established an NR-treated rheumatoid arthritis (RA) mouse model and classified the obtained metabolomic data using the Hessian-free SAE (HF-SAE) algorithm. During training, the unlabeled data were used for pretraining, and the labeled data were used for fine-tuning based on the HF algorithm for gradient descent optimization. The hybrid algorithm successfully classified the data. The results were compared with those of the support vector machine (SVM), *k*-nearest neighbor (KNN), and gradient descent SAE (GD-SAE) algorithms. A five-fold cross-validation was used to complete the classification experiment. In each fine-tuning process, the mean square error (MSE) and misclassification rates of the training and test data were recorded. We successfully established an NR animal model and an improved SAE for metabolomic data classification.

## 1. Introduction

Rheumatoid arthritis (RA) is a common systemic autoimmune disease characterized by symmetric polyarthritis and joint destruction [1]. It is traditionally treated with methotrexate combined with the botanical preparation of *Tripterygium wilfordii*. Good results are achieved with this treatment, which improves symptoms and delays disease progression. However, due to severe side effects, treatment compliance is poor. Naru3 (NR) is a traditional Mongolian medicine with a pure botanical preparation. Feng and Xiao [2] and Zhi [3] showed that the therapeutic effect of NR was similar to that of traditional RA treatment methods, and that it was a safe and effective drug of high medicinal value. However, the traditional Mongolian medicine (TMM) research methods are simplistic, and the technologies used are outdated. Therefore, it is necessary to combine these methods with modern technologies and approaches to further promote the application of TMM in disease diagnosis and treatment.

The article "An Improved Stacked Autoencoder for Metabolomic Data Classification" was published in 2021. Journal: Comput Intell Neurosci.

In recent years, machine learning and its subfield deep learning have been successfully applied in various fields, such as image processing, speech recognition, and natural language processing. Furthermore, they have attracted widespread attention in the fields of medicine, chemistry, and biology, exerting a great impact on people's life.

With the development of high-throughput experimental technologies, high-dimensional, noisy, and redundant biological or medical data can be obtained. However, owing to the cost of the experiments, the sample data are scarce, rendering the standard method of multiple regression inefficient. Assuming that *p* is the dimensionality and *n* is the amount of data, then *p* >> *n*. If we use limited data to build a distribution model with *p* parameters, it can easily lead to overfitting in machine learning models. This is a well-known problem in the field of statistics, known as the “curse of dimension” [4]. In the abovementioned research fields, there have been many successful applications of machine learning methods in solving the *p* >> *n* problem. Ueki and Tamiya have developed a new genetic prediction method using single nucleotide polymorphism (SNP) data in genome-wide association studies (GWASs), which has good predictive ability but is computationally expensive [5]. Ching et al. developed a new artificial neural network (ANN) framework, called Cox-nnet, to predict patient prognosis from high-throughput transcriptomic data, achieving the same or better predictive accuracy compared with that of other methods, including Cox-proportional hazards regression, random survival forests, and CoxBoost, while revealing richer biological information [6]. Xu et al. proposed a feature selection method for one-bit compressed sensing for the classification of high-throughput protein data based on mass spectrometry (MS), which has been employed on MS data to select important features with low dimensions, showing better classification performance for real MS data than traditional methods [7]. Yu et al. developed a support vector machine (SVM) algorithm that identifies optimal sorting gates based on machine learning using positive and negative control populations, taking advantage of more than two dimensions to enhance the ability to distinguish between populations [8]. Furthermore, Xie et al. proposed a RankComp algorithm, which was mainly developed to identify individual-level differentially expressed genes (DEGs) that can be applied to identify population-level DEGs for one-phenotype data [9]. Fouaz and Hacene proposed a genetic algorithm to improve similarity searching pertaining to ligand-based virtual screening, which can identify the most important and relevant characteristics of chemical compounds [10].

The article "An Improved Stacked Autoencoder for Metabolomic Data Classification" was published in 2021. Journal: Comput Intell Neurosci.

In recent years, metabolomic data processing has attracted increasing attention [11]. Metabolomics mainly studies how an organism's metabolites respond to changes in internal and external environmental conditions [12]. In metabolomics, a machine learning method is used to process data, screen biomarkers, and study the changes in metabolic pathways and the molecular mechanisms of diseases [13]. The analysis of metabolomic data is accompanied by multiple difficulties and challenges due to its high throughput, sparse, and high-dimensional nature and the *p* >> *n* problem [14, 15]. At present, although traditional machine learning methods such as principal component analysis (PCA) [16], random forest (RF) [17], and SVM [18] have been successfully applied in the field of metabolomics, it is still necessary to find better methods to process metabolomic data. Deep learning methods have been successfully applied in many fields but less in metabolomics [19]. A stacked autoencoder (SAE) is a typical deep learning model with good feature selection and nonlinear expression. An improved SAE algorithm needs to be developed to solve the problem of metabolomic data classification.

Although deep learning is a machine learning subfield with a wide range of applications, a limited number of deep learning-based metabolomic studies have been so far performed. Asakura et al. proposed an ensemble deep neural network (EDNN) algorithm, which they applied to metabolomic data of various fish species, that is helpful for regression analyses and concerns pertaining to classification in metabolomic studies. The dimensions of their experimental data were 106 and were derived from nuclear magnetic resonance (NMR) measurements [19]. Date and Kikuchi proposed an improved DNN-mean decrease accuracy (MDA) method that can be used for supervised classification and regression modeling and the determination of important variables for the evaluation of biological and environmental samples [20]. Alakwaa et al. proposed that metabolomics holds promise as a new technology for the diagnosis of highly heterogeneous diseases. However, it remains unknown whether DNN, a class of increasingly popular machine learning methods, is suitable for classifying metabolomic data. [21]. Bardley and Robert proposed that metabolomic data are complex because of their high dimensionality and high degree of multicollinearity between variables [22]. Risum and Bro successfully implemented a deep learning algorithm to perform automated spectral deconvolution [23]. Thus, it is reasonable to speculate that we are now within reach of a single deep learning algorithm for accurately classifying raw spectra directly from the instrument [24]. However, the limiting factor for success is to obtain sufficiently large datasets, which are required to train such computationally “greedy” algorithms [25].

The article "An Improved Stacked Autoencoder for Metabolomic Data Classification" was published in 2021. Journal: Comput Intell Neurosci.

Metabolomic data have a high throughput, sparse, high-dimensional, and small sample nature. Deep learning has good predictability, which shows that it can better distinguish different types of metabolomics data. If a good classification can be obtained, it will help us to further complete the selection of biomarkers based on deep learning. In this study, we aimed to introduce an improved framework, named Hessian-free [26] stacked autoencoder (HF-SAE), combining the Hessian-free algorithm and SAE model with Softmax regression for the classification of metabolomic data of NR-treated RA. We used this hybrid algorithm to perform the classification of metabolomic data of NR-treated RA and compared the results with those obtained using the SVM, *k*-nearest neighbor (KNN), and gradient descent SAE (GD-SAE) algorithms. A five-fold cross-validation was used to complete the classification experiment. In each fine-tuning process, the mean square error (MSE) and misclassification rates of the training data and test data were recorded. The hybrid algorithm successfully classified the data. A five-fold cross-validation was used to complete the classification experiment. In each fine-tuning process, the MSE and misclassification rates of the training and test data were recorded. We successfully established an NR animal model and an improved SAE for metabolomic data classification.

## 2. Methods

### 2.1. Metabolomic Stacked Autoencoder

The autoencoder was composed of an input layer, a hidden layer, and an output layer. The encoder encoded the input data, which were composed of an input layer and a hidden layer. The decoder completed the reconstruction of the input data, which consisted of a hidden layer and an output layer. Its purpose was to make the output as close as possible to the input. The training steps of the autoencoder were as follows.

#### 2.1.1. Calculation of the Activation Value of Each Layer

The sample data were the input of the encoder, and the activation value of the hidden layer neurons was calculated by forward conduction. The activation value of the hidden layer neurons was the input of the decoder, and its output (reconstruction value) was calculated in the same manner. If *f* (*z*) is used to represent the activation function, *a*_*i*_^*l*^=*f*(*z*_*i*_^*l*^) is the activation value of the i-th neuron in layer *l*.  *z*_*j*_^*l*+1^  represents the weighted sum of all inputs of the *j*-th neuron in the *l *+* *1 layer, and its formula is as follows:

(1) $$\begin{array}{c} z_{j}^{l+1}=\sum_{i=1}^{n}w_{ij}^{l}x+b_{j}^{l+1}, \end{array}$$

where *n* is the number of neurons in the *l* layer, *x* is the input. *w*_*ij*_^*l*^  is the weight between the *j*-th neuron of the *l *+* *1 layer and the *i*-th neuron of the *l* layer, and *b*_*j*_^*l*+1^  is the bias of the *jth* neuron in the *l *+* *1 layer.

The article "An Improved Stacked Autoencoder for Metabolomic Data Classification" was published in 2021. Journal: Comput Intell Neurosci.

#### 2.1.2. Updating Weights and Biases

The back-propagation (BP) was used to calculate the residual between each layer of neurons and the output layer, and BP was based on gradient descent to reduce the training error of the network. The cost function was used to calculate the least mean square error between the expected output and the actual output. *J* (*w*, *b*) is the cost function, and the formula is as follows:

(2) $$\begin{array}{c} J\left(w,b\right)=\frac{1}{m}\sum_{k=1}^{m}\left(\frac{1}{2}{\left\|a_{w,b}{\left(x\right)}^{k}-y^{k}\right\|}^{2}\right), \end{array}$$

where *m* is the number of samples, *x* is the input, *a*_*w*,*b*_(*x*)^*k*^  is the actual output, and *y* is the expected output. The error was used to adjust the weight and bias of the network based on BP so that the error was gradually reduced. Gradient descent was used to continuously update *w* and *b* so that the output of the autoencoder was close to the input. The adjusted value of *w* and *b* is proportional to ∂/∂*wJ*(*w*, *b*) and ∂/∂*bJ*(*w*, *b*). The formulas for updating *w* and *b* are as follows:

(3) $$\begin{array}{c} w=w-\alpha \frac{\partial }{\partial w}J\left(w,b\right),\\ b=b-\alpha \frac{\partial }{\partial b}J\left(w,b\right). \end{array}$$

#### 2.1.3. Activation Function

SAE is a deep neural network composed of multiple AE units. The model is trained layer by layer using an unsupervised method, and the output of the previous layer is the input of the next layer. The output of the SAE is the input of the classifier that completes the classification. The multihidden layer in SAE can effectively reduce the noise, improve the generalization ability, increase robustness, and improve the classification accuracy.

In the training, the restricted Boltzmann machine (RBM) was used to obtain the initial weight, and the ReLU was used as the activation function. A sigmoid is a common activation function that maps the output between [0, 1]. However, when the input values are close to infinity or infinitesimal, their gradient is close to zero. Therefore, it is very important to initialize the parameters. If the initial parameters are very small, most neurons are in the saturated state; that is, the gradient is close to 0, which makes the learning of the neural network extremely difficult. As mentioned above, ReLU was selected as the activation function of the SAE, and its formula was as follows:

(4) $$\begin{array}{c} a_{i}^{l}=f\left(z_{i}^{l}\right)=\max\left(0,z_{i}^{l}\right), \end{array}$$

where the gradient is always 1 when *z*_*i*_^*l*^* *>* *1, which indicates that the gradient is unsaturated. When the error is back-propagated, the update of the SAE weight can be completed quickly. Moreover, the calculation of ReLU is simple, and thus the running speed of the SAE is significantly improved.

The article "An Improved Stacked Autoencoder for Metabolomic Data Classification" was published in 2021. Journal: Comput Intell Neurosci.

### 2.2. Sparse Autoencoder

To better complete feature selection and reconstruction, the sparse method was used to limit the activity of neurons in the model. If *x* is the input of AE and *a*_*j*_^(2)^(*x*)  is the activation value of the hidden node *j*, the average activation value of the hidden node *j* is as follows:

(5) $$\begin{array}{c} {\hat{p}}_{j}=\frac{1}{m}\sum_{i=1}^{m}\left[a_{j}^{\left(2\right)}\left(x^{i}\right)\right], \end{array}$$

where *m* is the number of samples. In the sparse method, the penalty factor is added to the cost function of AE, and its formula is as follows:

(6) $$\begin{array}{c} \sum_{j=1}^{s_{2}}p\;\log\frac{p}{{\hat{p}}_{j}}+\left(1-p\right)\log\frac{1-p}{1-{\hat{p}}_{j}}, \end{array}$$

where *p* is a sparse parameter and its value is close to zero, $\hat{p_{j}}$ is determined by the connection weights and biases between the nodes of each layer, and *s*_*2*_ is the number of nodes in the hidden layer. We would like the average activation of each hidden neuron *j* to be close to zero. To achieve this, we add an extra penalty term to our optimization objective that penalizes ${\hat{p}}_{j}$deviating significantly from *p*. The optimized cost function of the sparse method is as follows:

(7) $$\begin{array}{c} J\left(w,b\right)=J\left(w,b\right)+\beta \sum_{j=1}^{s_{2}}p\;\log\frac{p}{{\hat{p}}_{j}}+\left(1-p\right)\log\frac{1-p}{1-{\hat{p}}_{j}}, \end{array}$$

where *β* is the weight of the sparse penalty factor.

### 2.3. Fine-Tuning

The proposed HF-SAE consists of SAE and Softmax regression. SAE completes feature selection, and Softmax regression completes the classification of metabolomic data. The structure of our neural network is 4573-1000-500-100-5, which includes three AE units and one Softmax unit. In the pretraining of the SAE, two adjacent layers formed an AE, and the connection weights between layers were obtained by AE training. The input of each AE hidden layer was the input of the next AE. In the process of fine-tuning, the entire SAE was considered as an encoder, and the mapping of the SAE was considered as a decoder. SAE and its mapping were combined into more hierarchical networks, and HF was used to fine-tune the weights. The fine-tuning structure is illustrated in Figure 1.

The article "An Improved Stacked Autoencoder for Metabolomic Data Classification" was published in 2021. Journal: Comput Intell Neurosci.

## 3. Results

### 3.1. Dataset

#### 3.1.1. Chemicals and Reagents

NR was provided by the Mongolian Medicine Manufacturing Room of the Affiliated Hospital of Mongolia University for the Nationalities (Tongliao, China). NR powder was dissolved in a 0.5% carboxymethyl cellulose (CMC) sodium aqueous solution up to a concentration of 1.00 g/mL and stored at 4°C for animal experimentation.

Radix *Aconiti kusnezoffii* (AK) and *Piper longum* (PL) were purchased from Liqun Drugstore (Tongliao, China). The AK and PL powders were refluxed eight times with ethanol for three times (2 h each time). The extraction solution was slightly boiled. After filtration, the concentrations of AK and PL supernatants were diluted to 0.28 and 0.17 g/mL, respectively.

Complete Freund's adjuvant (CFA) was purchased from Sigma Chemical Co. (St. Louis, MO, USA). Methanol and formic acid (Fisher Scientific, UK) were of HPLC grade. The assays were purchased from Nanjing Jiancheng Bioengineering Institute (Nanjing, China).

#### 3.1.2. Adjuvant-Induced Arthritis Model Establishment and Treatment

The study was approved by the ethics committee of the Medicine College of Inner Mongolia University for the Nationalities (IMUNMCEC20210412 [1]). Male Wistar rats (200 ± 10 g) were provided by YiSi Laboratory Animal Technology Co., Ltd. (Changchun, China). All animals were reared under standard conditions (21 ± 2°C, daily sunshine for 14 h) with free access to rodent chow and water in the Affiliated Hospital of Inner Mongolia University for Nationalities and allowed to acclimatize in metabolism cages for 1 week prior to the experiment. The rats were divided into five treatment groups: control (CG), model (MG), NR, AK, and PL, with eight rats in each group. On day 1, the rats in the MG NR, AK, and PL groups were intradermally injected with 0.1 mL CFA in the right posterior toe, while the rats in the CG group were injected with 0.1 mL saline. After 7 days, the rats in the MG, NR, AK, and PL groups were injected with 0.1 mL CFA. On day 14, the rats in the NR, AK, and PL groups were administered NR, AK, and PL, with the doses of 1.00, 0.28, and 0.17 g/kg/day, respectively, for 21 consecutive days, and on day 35 all the rats were euthanized. Blood was collected from the hepatic portal vein and centrifuged at 3500 rpm for 10 min at 4°C. The supernatants were immediately frozen, stored at −20°C, and thawed before analysis. Arthrodial cartilage was fixed in 10% formaldehyde for paraffin embedding.

The article "An Improved Stacked Autoencoder for Metabolomic Data Classification" was published in 2021. Journal: Comput Intell Neurosci.

#### 3.1.3. Serum Sample Preparation

The serum samples were thawed before analysis, and 100-*µ*L aliquots were added to 400 *µ*L acetonitrile, followed by vortexing for 30 s and centrifugation at 12000 rpm for 10 min at 4°C. The supernatant was subsequently filtered through a 0.22-*µ*m filter membrane.

#### 3.1.4. Ultrahigh-Performance Liquid Chromatography (UHPLC) Conditions

A Thermo Dionex Ultimate 3000 UHPLC system coupled with a *Q* Exactive Focus Orbitrap mass spectrometer (Thermo, USA) was used for metabolomic analysis.

The Waters Acquity UHPLC BEH C18 Column (1.7-*µ*m, 2.1 mm × 50 mm, Waters, UK) was maintained at 40°C with a flow rate of 0.3 mL/min^−1^ for the separation. The mobile phases were 0.1% formic acid in deionized water (A) and methanol (B). The gradient elution with B was performed according to the following schedule: 8% B for 0–0.5 min, 8–60% B for 0.5–1.5 min, 60–100% B for 1.5–6 min, 100% B for 6–8 min, 100–8% B for 8-9 min, and 8% B for 9-10 min. The sample injection volume was 10 *µ*L.

The optimal conditions used for UHPLC-high-definition MS (HDMS) analysis were as follows: nitrogen was used as the sheath and aux gas (at flow rates of 30 and 5 bar, respectively), the spray voltage was 3.0 kV, and capillary and aux gas heater temperatures were 320°C and 300°C, respectively.

The MS data were collected in switching mode (switching between positive and negative spectra) in the mass range of 100–1000 Da. The resolution of the full MS was 70000. In the dd-MS2 discovery mode, the resolution was 17500, and the isolation window was set to 3.0 m/z. The MS2 collision energy was set to 30 eV.

#### 3.1.5. Data Analysis

A pooled quality control (QC) sample was prepared by mixing aliquots (20 *µ*L) of each sample to monitor the instrument stability. Every day, six QC samples were analyzed to test the stability of the instrument. The Compound Discoverer software (version 2.0) was used for peak detection, alignment, and normalization of the peak area.

### 3.2. Five-Fold Cross-Validation Classification Experiment

The metabolomic dataset contained a small number of samples. To verify the reliability and stability of the HF-SAE model for classification, a five-fold cross-validation method was adopted. The data were divided into five groups on average. Each time, four groups were selected as the training set, and one group was selected as the validation set. The process was repeated until each group of data became a validation set.

The article "An Improved Stacked Autoencoder for Metabolomic Data Classification" was published in 2021. Journal: Comput Intell Neurosci.

We obtained 40 samples of metabolomic data from the NR-treated animal model. To better complete the training of the model, we used the synthetic minority oversampling technique (SMOTE) [27] algorithm to expand the experimental data to 320. There were 255 samples in the training set, 65 samples in the test set, and 4573 variables. The experimental data were preprocessed and normalized and divided into five groups (CG, MG, NR, AK, and PL). The structure of our neural network was 4573-1000-500-100-5. The learning rate was set to 0.01. First, the unsupervised method was used to complete the SAE training (the pretraining of the model was completed, and the initial weight was obtained). Second, a supervised method was used to complete the training of the Softmax classifier. Finally, fine-tuning of the model was completed, in which the GD and HF algorithms were used to minimize the cost function. Owing to the small number of training and test data, a min-batch was not used in the training process. The number of iterations in each RBM during training was 500, and the number of iterations during fine-tuning was 4000. The classification accuracies are presented in Table 1.

Table 1 shows the results of the five-fold cross-validation classification experiment for the different datasets. The KNN classification accuracy was between 81.54% and 86.15%, with the lowest accuracy being observed in the third group. The SVM classification accuracy fluctuated dramatically between 73.85% and 81.54%, with the lowest accuracy being observed in the first group. When we used the method combining SAE with Softmax regression, in which fine-tuning was based on GD or HF, the GD-SAE classification accuracy was between 70.77% and 76.92%, and that of HF-SAE was over 90% for each group and did not fluctuate dramatically. The SVM classification accuracy varied greatly and lacked robustness. Although the classification results of KNN and GD-SAE were stable, the classification accuracies were not satisfactory. Therefore, the proposed method is more stable, reliable, and suitable for the classification of metabolomic data. To further compare the effects of different fine-tuning algorithms on the SAE, we recorded the MSE of the training set and the misclassification rate of the training and test sets. A comparison of MSE, training, and test classification error rates is shown in Figure 2.

For terms of the running time, KNN, SVM, GD-SAE, and HF-SAE were about 80 seconds, 80 seconds, 650 seconds, and 900 seconds, respectively. Although HF-SAE had a good classification effect, the computational complexity was very high. In addition, we also evaluated the classification accuracy by calculating the kappa value [28], and the range of this value is [0, 1]. If the value was closer to 1, it indicated that the classification accuracy of the model was better. The kappa value of KNN, SVM, GD-SAE, and HF-SAE was 0.81, 0.72, 0.68, and 0.91, respectively. The proposed HF-SAE method had the best kappa value, which further showed that the method had better classification ability.

The article "An Improved Stacked Autoencoder for Metabolomic Data Classification" was published in 2021. Journal: Comput Intell Neurosci.

### 3.3. Classification Experiments of Different Training and Test Datasets

Metabolomic data have a high throughput, sparse, high-dimensional, and small sample nature, which increases the classification difficulty. To further verify the effect of different methods on metabolomic data classification, six datasets with different sizes were established, and the data content difference between each group was 10%. The experiment algorithm was the same as that used in the five-fold cross-validation classification experiment. The number of training sets and test sets for each group, as well as the classification results, is listed in Table 2.

Table 2 shows that when the training data decrease with the decrease in total samples, the classification accuracy of KNN, GD-SAE, and HF-SAE also significantly declines. The reason is that the above three machine learning methods are affected by the reduction of the features that can be obtained, while the accuracy of SVM is relatively stable and less affected by this. Compared with the other three methods, HF-SAE can provide better results. In metabolomic data classification experiments of different scales, it is shown that although the training data are reduced, HF-SAE can still obtain better metabolomic data characteristics.

## 4. Discussion

In the five-fold cross-validation classification experiment, the GD-SAE average classification accuracy rate was the lowest, while that of HF-SAE was the highest. The experimental results show that if the fine-tuning methods of the SAE classification model are different, the effect on the results is very obvious. As the number of iterations increased, the fine-tuning process differed significantly. To further compare the effects of different fine-tuning algorithms on the SAE, we recorded the MSE of the training set and the misclassification rate of the training and test sets. In the five-fold cross-validation experiment based on the GD fine-tuning method, the MSE decreased slowly with the increase in iteration, and the misclassification rate of the training and test sets also gradually decreased during the oscillation process. However, this downward trend was not obvious. When the iteration reached a certain number of times, only a certain range of oscillation occurred, but there was no trend of continuous decline. In the five-fold cross-validation experiment based on the HF fine-tuning method, each indicator had a fast decline speed and small amplitude, and fewer iterations were needed to reach a stable interval compared with GD.

The article "An Improved Stacked Autoencoder for Metabolomic Data Classification" was published in 2021. Journal: Comput Intell Neurosci.

In the process of fine-tuning, the classification accuracy of GD and HF tended to be stable after 2000 iterations, but their classification effect was obviously different. This shows that GD only reaches the local optimal state during fine-tuning and cannot jump out of the local minimum. The change in MSE also explains the difference in the classification accuracy. The MSE of the HF showed a clear downward trend and stabilized after approximately 2000 iterations. Although the GD showed a downward trend, the change was small. The HF-SAE proposed in this paper is superior to the GD-SAE in both the classification results and the fine-tuning process. Moreover, the HF-SAE is stable, reliable, and suitable for metabolomic data classification. A comparison of MSE, training, and test classification error rates is shown in Figure 2. For terms of the running time, KNN was the shortest, HF-SAE time was the longest, and the computational complexity was the highest. HF-SAE achieved better classification results at the cost of consuming more computing resources.

In the classification experiments of different training and test datasets, the number of fine-tuning iterations was 4000. The training data for the experiment were reduced from 255 to 128, and the test data were reduced from 65 to 32. In each group of experiments, the classification result of HF-SAE was better than that of GD-SAE. In the fine-tuning process, the HF-SAE error rate amplitude was relatively large in the initial stage. The classification error rate decreased faster and entered a stable and small-amplitude oscillation range in a short time. The GD-SAE classification accuracy only showed a significant decline in the initial stage of fine-tuning. However, there was no significant change in the classification accuracy, which was significantly different from the classification results of HF-SAE.

In the method comparison, accuracies of HF-SAE were superior for the classification of metabolomic data of NR-treated RA compared with KNN, SVM, and GD-SAE. Accompanying development of metabolomics, robust and accurate classification methods to predict sample labels are in critical need. These results indicated that the HF-SAE developed here was a helpful tool for analyzing biomarkers from the metabolomic data. We concluded that the HF-SAE was capable of identifying important variables that contributed to the constructed HF-SAE model.

Although HF-SAE has excellent classification performance, there are still some considerations in metabonomics research. Compared with some other machine learning methods, HF-SAE is time-consuming computation. In addition, metabonomics datasets are typically small compared with other data, such as text and images. For the classification of metabolomic data of NR-treated RA, we obtained 40 samples. To better complete the training of the model, we used the SMOTE algorithm to expand the experimental data to 320 because very small data sets may not be suitable for HF-SAE. We also experimented with the effects of reducing training set size and test set size and found that HF-SAE is indeed sensitive to the sample size of the study.

The article "An Improved Stacked Autoencoder for Metabolomic Data Classification" was published in 2021. Journal: Comput Intell Neurosci.

## 5. Conclusions

NR is a traditional Mongolian medicine and a pure botanical preparation, and it has achieved good results in improving symptoms and delaying RA progression. However, the TMM research methods are simplistic, and the technologies used are outdated. Therefore, HF-SAE was used to classify the metabolomic data of NR-treated RA. Metabolomic data are highly dimensional and sparse. With the proposed method, we not only diagnosed RA but also completed an evaluation of NR. In the five-fold cross-validation classification experiment, the proposed method is more stable, reliable, and suitable for the classification of metabolomic data compared with KNN, SVM, and GD-SAE. To further verify the effect of different methods on metabolomic data classification, we performed classification experiments using different training and test datasets. The results show that although the training data are reduced, HF-SAE can still obtain better metabolomic data characteristics. Although the HF-SAE algorithm is a useful tool for the classification, the performance of the method depends on sample size, and how to select biomarkers and explain the model scientifically through the model proposed is also an urgent problem to be solved in this field at this stage.

## Figures and Tables

**Figure 1:** Fine-tuning structure (SAE, stacked autoencoder).

**Figure 2:** Fine-tuning of experimental results on the five-fold data sets. The red and blue lines represent the GD-SAE and HF-SAE results, respectively. In each subgraph of (a) to (e), (i) shows the FMSE, (ii) shows the CR of the training set, and (iii) shows the CR of the test set (GD-SAE, gradient descent stacked autoencoder; HF-SAE, Hessian-free SAE; FMSE, fine-tuning mean square error; CR, classification rate).

**Table 1:** Classification accuracy in the five-fold cross-validation experiment (%).

Group	KNN	SVM	GD-SAE	HF-SAE
1	84.62	73.85	70.77	93.85
2	86.15	76.92	76.92	92.31
3	81.54	81.54	73.85	90.77
4	84.62	75.38	75.38	93.85
5	87.69	78.46	73.85	93.85
Mean	84.92	77.23	74.15	92.93

The article "An Improved Stacked Autoencoder for Metabolomic Data Classification" was published in 2021. Journal: Comput Intell Neurosci.

**Table 2:** Classification accuracies of the different training and test sets (%).

Training set	Test set	KNN	SVM	GD-SAE	HF-SAE
255	65	86.15	76.92	76.92	92.31
230	58	82.76	84.48	77.59	91.38
204	52	80.77	80.77	76.92	88.46
179	45	77.78	75.56	77.78	84.44
153	39	76.92	79.49	74.36	84.62
128	32	71.88	78.13	68.75	81.25

## Data Availability

Our data still need to be studied in the next stage, so it is not convenient to provide it directly. The data can be made available upon request via email.
